# An Individual Driving Behavior Portrait Approach for Professional Driver of HDVs with Naturalistic Driving Data

**DOI:** 10.1155/2022/3970571

**Published:** 2022-01-22

**Authors:** Yi He, Shuo Yang, Xiao Zhou, Xiao-Yun Lu

**Affiliations:** ^1^Intelligent Transport Systems Research Center, Wuhan University of Technology, Wuhan 430063, China; ^2^CATARC (Tianjin) Automotive Information Consulting Co., Ltd., Beijing 100011, China; ^3^School of Mechanical and Electronic Engineering, Wuhan University of Technology, Wuhan 430063, China; ^4^California PATH, University of California, Berkeley, CA 94804-4684, USA

## Abstract

More than 50% major road accidents are caused by risk driving behaviors from professional drivers of Heavy Duty Vehicles (HDVs). The quantitative estimation of driving performance and driving behaviors portrait for professional drivers is helpful to measure the driver's driving risk and inherent driving style. Previous studies have attempted to evaluate risk driving behavior, but most of them rely on high-demand vehicle and driving data. However, few studies can dig into the causes and correlations behind individual driving behavior and quantify the driving behaviors portrait for professional driver based on long-term naturalistic driving. In this study, the data is from On-Board Unit (OBU) devices mounted in the HDVs in China. Based on the driving behavior pattern diagram and the frequency and ranking of drivers' typical driving patterns, a driving behavior portrait approach is proposed by comprehensively considering the vehicle safety, driving comfort, and fuel economy indicators. The similarities and differences of different drivers' driving behaviors are quantitatively analyzed. The high precision and sampling frequency data from vehicles are used to verify the proposed approach. The results demonstrated that the driving behavior portrait approach can digitally describe the individual driving behaviors styles and identify the potential driving behaviors with long-term naturalistic driving data. The development of this approach can help quantitatively evaluate the individual characteristic of risk driving behaviors to prevent road accidents.

## 1. Introduction

More than 50% major road accidents are caused by risk driving behaviors from professional drivers of HDVs [1]. Due to drivers' personal characteristic and driving style, most of the road accidents are caused by risk driving behaviors [2]. Quantifying analysis drivers' driving style and identifying driving behavior portrait is helpful to prevent road accidents.

In recent years, many studies have attempted to evaluate risk driving behavior, but most of them rely on high-demand vehicle and driving data, which is not conducive to large-scale application, and most of the previous studies focus on driving safety levels or identify the driving behaviors based on real time or offline with short-term data analysis ([3–12]; Yan et al., 2019). However, few studies can dig into the causes and correlations behind individual driving behavior and quantify the driving behaviors portrait for professional driver based on long-term naturalistic driving.

Various driving behaviors can be seen as the responses to complex driving conditions. Due to the personal characteristics and driving skills of different drivers, their driving behaviors are also different. Some drivers have aggressive driving styles, fast acceleration, and braking with high risk driving, while others are more cautious with less risk. Therefore, the quantitative estimation of driving performance and driving behaviors portrait is helpful to measure the driver's driving risk and inherent driving style, so as to prevent traffic accidents.

With the development of autonomous and connected vehicle, various sensors can be installed on the vehicle to collect real time data with naturalistic driving. However, the positioning data is the most widely used and has high precision with large-scale application in real traffic until now.

In this paper, the data is from OBD devices mounted in the HDVs in China, and high precision and sampling frequency data from vehicles are used to verify the proposed approach. Based on the driving behavior pattern diagram and the frequency and ranking of drivers' typical driving patterns, a driving behavior portrait approach is proposed by comprehensive considering the vehicle safety, driving comfort, and fuel economy indicators, to quantitatively evaluate the personalized driving behavior of different drivers and identify potential risk driving behaviors, so as to improve the assessment accuracy of the risk model and reduce the accident risk.

## 2. Literature Review

The majority of road accidents are caused by risk driving behaviors of professional drivers with HDVs. Therefore, scholars from all parties have carried out assessment studies on drivers' driving safety and driving risk, mainly from the following three aspects.

### 2.1. Risk Driving Behavior Identification Based on Statistical Methods

Some risk driving behavior studies are related by applying statistical method or machine learning algorithm to classify and identify risk driving. Constantinescu et al. modeled driving styles based on positioning data and divided drivers into different driving styles by cluster analysis and principal component analysis [8]. Suzdaleva et al. studied the stochastic modeling of driving style and its online estimation during driving based on Bayesian theory, and their research used recursive algorithm to estimate hybrid parameters and actual driving style [7]. Martinez et al. introduced a vehicle driving style feature and recognition correction algorithm based on current and future development trends with machine learning methods [9]. Qi et al. studied two thematic models: mLDA and mHLDA, which can discover the information of differentiated driving styles with hidden structures from the data of real driving behaviors and can identify the different driving styles [10]. Zhu et al. proposed an unsupervised clustering algorithm that can reflect different driving styles [13]. Han et al. proposed a method of driver behavior uncertainty identification based on statistics [11]. Wang et al. used semisupervised support vector machines to classify driving styles. In order to solve the problem that supervised learning method requires a large amount of marked training data and it is time-consuming to manually label a large amount of driving data, a semisupervised support vector machine method is used in this paper to classify drivers into aggressive driving style and conventional driving style according to several marked data points [6]. Siordia et al. proposed an autonomous driving risk rating system. The system is based on a driving simulator that uses driver, road, and vehicle information to train five different data mining algorithms to predict the level of driving risk [14].

### 2.2. Risk Driving Behavior Identification Based on Safety-Related Driving Events Detection

Another commonly used method for classifying driving risks is to detect safety-related driving events, such as sharp acceleration, sharp deceleration, and sharp turns. In Johnson et al.'s study, a dynamic time structuring algorithm (DTW) was used to detect the driving styles with data from smartphone sensors [15]. In this case, they need some predefined templates for the detected driving events. Itkonen has made a trade-off between the compact but erratic behavior of driving and the loose and smooth following behavior of driving. They call it “tight” and “smooth” driving and suggest that this trade-off can be used as a potential factor to evaluate potential driving styles [16]. In these studies, the use of predefined driving events is essential, but the thresholds used to define these driving events are not consistent. For example, in Paefgen et al.'s study, the threshold value used for rapid acceleration and deceleration is ±0.1 g [17]. Fazeen uses ±0.3 g [3]. Wang et al. proposed a self-designed driving style scale, which is suitable for evaluating the driving style of drivers with Chinese national conditions [18]. Bagdadi proposed a method based on critical jerk, to identify safety critical braking events during car driving [19]. Chen et al. proposed a method to predict risk driving events and defined risk driving events by using the risk attribute diagram (ARM) [4].

### 2.3. Risk Driving Behavior Identification Based on Risk Modeling

Some scholars have also modeled the safety of drivers' driving behavior. Ellison et al. assessed the risk driving behavior by modeling driver behavior. The frequency and size of overspeed event, aggressive acceleration event, and aggressive braking event were used as the behavior measurement indexes, and their spatial and temporal characteristics were used as the influencing factors. Based on these parameters, the behavioral characteristics of drivers were established and the total score representing driving risk was given [5]. Bejani et al. developed the system to consider the impact of traffic levels and vehicle types on driving style assessments. The system consists of three subsystems, which use smart phones for calibration, driving action classification, and driving style evaluation [20]. Hong et al. used sensors such as Android smartphones, On-Board Diagnostics (OBD), and Inertial Measurement Units (IMU). By collecting driving behavior characteristics such as maximum speed and acceleration, average value, and standard difference, the relationship between driving characteristics and driving style was modeled by using naive Bayes classifier [21]. Jachimczyk et al. proposed a method to objectively evaluate driving style based on eight indexes related to speed, acceleration, engine speed, and driving time. This method is an embedded system based on the conceptual design of the Internet of things to evaluate three driving style standards: safety, economy, and comfort [22]. Meseguer et al. designed an Android application that can monitor physiological data from drivers and diagnostic data from vehicles in real time to study the correlation between heart rate and driving style [23]. Chu et al. proposed an improved curve speed model that takes into account driving style, vehicle, and road factors. On the basis of vehicle-road interaction model, driver behavior factor is introduced to quantify the driving style selected for the speed of curve [12, 24]. Deng et al., in order to identify driving styles, reasonably modeled three driving styles (aggressive, moderate, and mild) by means of hidden Markov model according to the driver's braking characteristics and realized efficient analysis of driving styles [25]. An early warning system has been proposed for risk driving based on statistical modeling. They used a semisupervised learning method to grade the driving risk and evaluate the safety of the driving time series data [26].

In summary, most of the risk driving behaviors studies focus on the classification of driving styles or the scoring of risk driving behaviors. The purpose of these previous studies is mostly to classify drivers into different driving safety levels, such as safe, normal, or dangerous, and rarely pay attention to individual driving behavior characteristics. In addition, the use of predefined risk driving behaviors models or events is essential, but the thresholds used to define these driving events are not consistent. However, a few studies focusing on the risk driving behavior model for professional driver of HDVs and a fixed risk driving threshold may not fit in all drivers due to various driving styles from individual drivers and understanding of the driving skills and experience.

In recent years, Internet portrait technology is widely used to quantify the characteristics of users. A driving habit graph (DHG) was proposed to model driving behaviors graphical model [4], which can quantify the behaviors parameters in naturalistic driving data and visual presentation of driving behaviors. Inspired by that study, this paper proposes an individual driving behavior portrait by comprehensively considering the vehicle safety, driving comfort, and fuel economy indicators to quantify the potential risk driving behaviors and driving styles.

## 3. Methodology

### 3.1. Driving Behavior Pattern Diagram

Driving behavior is the driver's response to different driving situations, and driving behavior patterns reflect these continuous driving behaviors over time; in this case, each driver has individual typical driving mode. We need to identify these driving behavior patterns and extract the representative ones to judge the driver's driving style based on the driving patterns of different drivers to evaluate the driver's driving safety level. In the process of method exploration, we use the Symbol Aggregation Approximation (SAX) method to convert the original driving data into the corresponding driving acceleration level code to reduce the complexity of original driving data [27]. SAX algorithm was proposed by Lin et al. in 2003 [28]. Based on the Piecewise Aggregation Approximation (PAA) method, this method retains its advantages of simplicity and low complexity and provides high sensitivity and selectivity in the process of range query. In addition, the symbolic feature representation provides a favorable condition for the existing rich data structures and string processing algorithms. The SAX process consists of two steps. First, convert the original data into a segmented aggregation approximation (PAA) representation. Second, convert PAA data to the corresponding string according to the location of the breakpoint. In this study, the driving behavior data was ultimately converted into a numeric code rather than a string. This research includes four steps: data standardization, data grading and coding, typical driving behavior pattern extraction, and driving behavior pattern graph generation.

#### 3.1.1. Data Standardization

In this study, the longitudinal acceleration change of the driver is used as the standard to reflect the driving behavior. Longitudinal acceleration is chosen as the standard because acceleration is a typical index closely related to driving safety, and the change of acceleration also represents the change of speed, which is another important index of driving safety.

The driving acceleration data of a certain driver is standardized by *Z*-standardization method, so that its mean value is 0 and the standard deviation is 1. The purpose of this is to make the offset and amplitude consistent so that it has the same dimension as other driver data.

#### 3.1.2. Data Grading and Coding

The grading and encoding of data require the use of SAX method. The SAX method first converts the original data into PAA representation. The PAA data is then converted to the appropriate string based on the location of the breakpoint.

This study divided the data into 7 levels. Theoretically, the SAX method can divide the data into up to 20 levels and provide corresponding thresholds. Based on data analysis, after testing the classification of 3, 5, 7, 9, and 11 grades, we found that the classification of 7 grades had the best effect. Only the odd number level is tested because the median level always represents a neutral behavior. In this study, the median represents the driving behavior of the vehicle approaching uniform cruising speed. Since the mean of the normalized data is 0, level 3 represents neutral behavior. Taking the acceleration data as an example, level 3 represents the acceleration value close to 0 m/s^2^, that is, uniform speed cruising. Levels 0, 1, and 2 represent negative acceleration, or deceleration. The amplitude range of data values for each level increases as the level decreases. As the number of levels decreases, the deceleration behavior becomes more obvious. Levels 4, 5, and 6 represent positive accelerations, or accelerations. The amplitude range of data values for each level increases with the level. As the rank value increases, the accelerating behavior becomes more obvious.

#### 3.1.3. Typical Driving Behavior Pattern Extraction

After the data is graded and coded, the driving mode that exists in it needs to be detected. Driving is a continuous process in which the vehicle is controlled by the driver's constant adjustment to achieve the desired driving condition. Limited by people's physiological and psychological factors, the reaction speed of the driver to the stimulus is limited. Under general conditions, the reaction time for complex selective reactions is 1∼3 s, and the reaction time for complex judgment and recognition is 3∼5 s on average. Studies have shown that three seconds is a window of time to measure driving behavior, during which the driver can adjust the vehicle to the desired state. Thus, the driving mode is defined as a change in driving behavior (speed, acceleration, steering, etc.) every three seconds. To make sure the timing is right, this article also tested using 4, 5, and 6 seconds. The results show that if these intervals are used as the detection time, a large number of driving mode types are generated, and the graph is not as clear as the result of 3 seconds. Starting from the starting point of the data, a moving window of window size 3 s is used to detect the existing driving mode. Due to the differences in driving skills and personal characteristics, each driver has his own unique driving habits. According to all the driving behavior patterns detected by different drivers, the driving behavior patterns with high frequency are used to represent the driving habits of drivers. For each driver, more frequent driving behavior patterns, that is, typical driving behavior patterns, were extracted. Driving patterns with the same sequence of combinations naturally converge into a group and count the number of patterns contained in each group. Then, the incidence of each driving behavior pattern was calculated. For example, if driving mode “123” occurs “*m*” times in a continuous acceleration data set of length “*n*,” the incidence of driving behavior mode “123” is “*m*/(*n* − 2)”. For each driver, the 30 most frequent driving behavior patterns were extracted and regarded as their typical driving behavior patterns. On the premise of collecting enough driving data to cover various external factors such as traffic conditions and road types, these typical driving behavior patterns can describe drivers' internal driving habits. In addition, these typical driving behavior patterns are independent of external driving conditions and reflect drivers' inherent driving preferences.

#### 3.1.4. Driving Behavior Pattern Graph Generation

The typical driving patterns were plotted in descending order of frequency to obtain the driving behavior pattern of individual drivers. Driving behavior data can be transformed into a graph through the four steps described above. The typical driving behavior pattern reflects the driver's personalized driving behavior, but also includes the driver's driving styles and hidden driving risks. In this study, the driving behavior patterns of drivers were plotted based on the acceleration data. For all driving behaviors, the first 30 driving patterns are extracted as the typical driving patterns. These 30 patterns are enough to reflect the driver's driving behavior characteristics. In addition, considering that acceleration and deceleration are two important and independent operations, the typical driving patterns of acceleration and deceleration are extracted, respectively, to illustrate the driving behavior characteristics of drivers and distinguish the differences between drivers' driving styles.

The abscissa in Figure 1 represents the first 30 typical driving behavior patterns that appear from high to low frequency after the extraction of typical driving patterns. The ordinate represents the seven acceleration levels of 0–6 after data classification and coding. That is, the combination of every three connected line points in the figure is a typical driving behavior pattern, and the corresponding abscissa is the occurrence frequency ranking of the behavior pattern, while the ordinate represents the corresponding acceleration level change of the driving behavior pattern within three seconds. Acceleration level 3 represents the neutral behavior, which is close to the acceleration value of 0 m/s^2^, that is, the average speed of travel. Acceleration levels 0, 1, and 2 represent the negative acceleration value, that is, the deceleration behavior. The amplitude range of data values for each level increases as the level decreases. As the number of levels decreases, the deceleration behavior becomes more obvious. The acceleration levels of 4, 5, and 6 represent the positive acceleration value, that is, the acceleration behavior. The amplitude range of data values for each level increases with the level. As the rank value increases, the accelerating behavior becomes more obvious. Taking the first typical driving behavior pattern “333” as an example, the frequency of this pattern is the highest. During the duration of this behavior pattern, the driver's acceleration level changes to “3-3-3.” The second driving behavior pattern, “343,” was the second most frequent. During the 3 seconds of this behavior pattern, the driver's acceleration level changed to “3-4-3.” The driver's driving behavior pattern diagram can clearly present the composition and sequence of the driver's typical driving behavior pattern.

### 3.2. Modeling Driving Behavior Risk

The driving behavior pattern graph is the visual representation and qualitative description of the driver's driving pattern. However, the frequency and ranking of typical driving patterns and the gradation of the patterns themselves offer possibilities for quantitative analysis. Therefore, taking acceleration data and typical driving patterns as influencing factors, this paper proposes a personalized driving behavior evaluation model from three aspects of vehicle safety, driving comfort, and fuel economy to comprehensively evaluate vehicle driving safety.

(1) $$\begin{array}{c} \begin{array}{c} \text{SCORE}=0.7*{\text{score}}_{\text{safe}}+0.2*{\text{score}}_{\text{comfort}}+0.1*{\text{score}}_{\text{economy}} \end{array}. \end{array}$$

As shown in formula (1), SCORE is the comprehensive evaluation index of driving behavior, which consists of three parts. The first part is the safety evaluation index based on the driver's typical driving behavior, which reflects the driver's driving safety degree and the severity of acceleration and deceleration. The second part is the evaluation and analysis of vehicle comfort based on acceleration data, which reflects the degree of comfort in driving behavior to some extent. The third part is the evaluation index of fuel economy based on acceleration, which reflects the degree of fuel consumption. Combined with literature, considering the operation of the vehicle in the process of driving safety is most important, followed by the comfort in the process of transportation, and finally to fuel economy, giving three sections of the score to the corresponding proportion of weight (i.e., safety weight with 70%, comfort with 20%, and the economy with 10%), comprehensive comparing to the driver's driving behavior evaluation.

(2) $$\begin{array}{c} \begin{array}{c} {\text{score}}_{\text{safe}}=\overset{30}{\underset{i=1}{\sum }}{\text{freq}}_{i}*\left\{\text{abs}\left[\text{mean}\left(\text{CODE}\right)-3\right]+\text{ std}\left(\text{CODE}\right)\right\} \end{array}. \end{array}$$

As shown in formula (2), in the first part, *i* is the order of the typical driving mode, and freq_*i*_ is the proportion of the typical driving pattern in all driving patterns. CODE is the code for a typical driving pattern, such as “234.” Mean and std were used to calculate the mean and standard deviation of driving patterns, respectively. For example, the mean of pattern “234” is (2 + 3 + 4)/3 = 3, and the standard deviation is 1. Abs stands for absolute value. This evaluation method can reflect the degree of safety of driving behavior, because it takes into account the amplitude and variation of acceleration value by using the mean value and standard deviation. The amplitude of driving acceleration and the change of acceleration are important indexes, so the mean value and standard deviation are added. In abs [means (CODE) − 3], −3 is the acceleration amplitude used to evaluate acceleration and deceleration behavior, because CODE 3 represents uniform driving behavior. This quantitative analysis method can consider the amplitude and change of acceleration at the same time, which can reflect the change of vehicle state and the change of vehicle control stability. Clearly, lower scores mean safer driving behavior.

(3) $$\begin{array}{c} \begin{array}{c} {\text{score}}_{\text{comfort}}={\left[\frac{1}{T}\int_{0}^{T}a_{w}^{2}\left(t\right)\text{d}t\right]}^{1/2} \end{array}. \end{array}$$

In the second part, score_comfort_ represents the root mean square value of weighted acceleration. *T* is the period (*s*) of vibration analysis; *a*_*w*_ (*t*) is the axial acceleration (m/s^2^); time history *a* (*t*) is the time history of weighted acceleration obtained by the weighted function filter *w*(*f*) of the corresponding frequency. This method refers to the evaluation standard of vehicle comfort formulated by ISO and only considers the influence of longitudinal acceleration on vehicle comfort. Lower scores mean a more comfortable driving.

(4) $$\begin{array}{c} {\text{score}}_{\text{economy}}=\left\{\begin{array}{c} {\text{MOE}}_{e}=e^{\sum_{i=0}^{3}\sum_{j=0}^{3}\left(L_{i,j}^{e}*v^{i}*a^{j}\right),a\geq 0},\\ {\text{MOE}}_{e}=e^{\sum_{i=0}^{3}\sum_{j=0}^{3}\left(M_{i,j}^{e}*v^{i}*a^{j}\right),a<0}. \end{array}\right. \end{array}$$

In the third part, score_economy_ represents the fuel consumption of the vehicle. Here, VT-Micro fuel consumption model proposed by Virginia Tech University is adopted. This method can be used to calculate instantaneous fuel consumption based on vehicle speed and acceleration, and it is proved that the model results have a high degree of fit with the actual fuel consumption, where MOE_*e*_ is the instantaneous fuel consumption (*L*/*s*) of the vehicle;  *v* is the instantaneous speed of the vehicle (km/h); *A* is the instantaneous acceleration of the vehicle (km/h/s); *L*_*i*,*j*_^*e*^ is the fitting coefficient of the instantaneous fuel consumption model when the vehicle is accelerating; the power of velocity *v* is *i* and the power of acceleration is *j*. *M*_*i*,*j*_^*e*^ is the fitting coefficient of the instantaneous fuel consumption model when the vehicle slows down and the power of velocity *v* is *i* and the power of acceleration is *j*. The fitting coefficient can be obtained by querying the coefficient value table of the model. Lower scores for this segment mean more economical fuel consumption for vehicles. It should be noted that the overall driving behavior evaluation score consists of three evaluation index scores, and these evaluation indexes have different orders of magnitude and dimensions. If the original index data value is directly used for summation analysis, the results are easy to be unreliable; that is, the index with higher value will be highlighted, while the index with lower value level will be weakened. Therefore, the scores of different indicators need to be standardized.

## 4. Driving Behavior Characteristics and Risk Analysis

### 4.1. Acquisition of Experimental Data

The data used in this paper was collected by the information acquisition equipment installed on the HDVs. The collection device includes a GPS module for collecting location data, an OBU module for collecting vehicle movement data, and a cellular network module for uploading the collected data to a server. The collected information is uploaded to the Internet of vehicles service platform in real time. The parameters collected include the vehicle's GPS time, speed, direction, mileage, position, longitude, latitude, ACC state, and positioning state, etc. The data sampling frequency is 1 Hz.

The natural driving data of 10 HDVs were collected, including driving behavior data. The driving environment of these experimental vehicles includes different grades of roads such as highway, national highway, provincial highway, county highway, and rural highway. The professional drivers are generally older and the average daily driving distance of vehicles is more than 100 kilometers. There is a one-to-one correspondence between the driver and the vehicle. Data collection period is from June 29, 2019, to July 29, 2019, a total of 30 days; more than 6 million pieces of driving data are collected. The drivers in the experiment did not have fixed working hours or rest days, and most of them drove during the day. The working period was from 7:00 AM to 17:00 PM. The data collection time was long enough and of high quality to reflect the driving behavior of individual drivers and meet the needs of the experiment.

For the practicality of the proposed approach in real life, meanwhile, considering the positioning data is the most widely used and has high precision with large-scale application in real traffic until now; in addition, the acceleration is a typical index closely related to driving safety; the change of acceleration also represents the change of speed, which is another important index of driving safety. Therefore, in the analysis of driving behavior, this study mainly uses the longitudinal acceleration data of drivers.

### 4.2. Driving Safety Preassessment

Before analyzing the driving behavior pattern, this study needs to make a prejudgment on the driving situation of individual drivers, that is, to preliminarily evaluate driving safety by identifying the frequency of risk driving events. In this paper, two risk driving behaviors of sharp acceleration and sharp deceleration are considered, and the acceleration threshold value of ±0.3 g proposed by Fazeen in this paper is used to detect these two driving behaviors. Using these thresholds, a quantified scoring method was used to assign each driver a driving safety label. Firstly, the proportion (percentage) of individual drivers' accelerated driving behavior (acceleration greater than 3 m/s^2^) and decelerated driving behavior (acceleration less than −3 m/s^2^) in the total driving behavior was calculated. The total proportion of drivers is high, indicating that the driver operates frequently with rapid acceleration and has relatively low safety in driving behavior. The evaluation results are shown in Figure 2.

As can be seen from Figure 2, the accelerated or decelerated behaviors of different drivers account for a low proportion of all driving behaviors. The proportion of rapid deceleration behavior of most drivers is higher than that of rapid acceleration behavior. The proportion of acceleration behavior and deceleration behavior of different drivers conforms to the same trend. The driver with a high proportion of risk driving behavior has a tendency of more risk driving behavior. For example, the driver Q01868D has a higher proportion of accelerated behavior than other drivers. However, drivers with a low proportion of risk driving behaviors can temporarily consider their driving behaviors to be relatively safe, such as D41777 and D41981. In order to facilitate the subsequent comparative analysis, we divided the ten drivers into two groups. Assume that the top 5 with the highest proportion of total behaviors of rapid acceleration and deceleration include B32781, B32791, B66980, F63022, and Q01868D as drivers in the relatively dangerous group. The 5 drivers with a low proportion of rapid acceleration and deceleration behavior, including B67845, D41777, D41981, D46109, and F63030, were taken as the drivers in the relative safety group. The following will explore the personalized driving styles of different drivers more specifically by analyzing the driving behavior pattern.

### 4.3. Integrated Driving Behaviors

As can be seen from Figures 3 and 4, the most frequent driving behavior pattern of all drivers was cruising “333.” The driving behavior pattern of individual drivers can clearly understand the driving styles of different drivers and their behavioral preferences in some driving situations. The shape and distribution of driving patterns can reflect the driving behavior characteristics of drivers, such as D41981 and Q01868D. The degree of dispersion and fluctuation of the driving behavior pattern of the two drivers can obviously reflect the degree of driving aggressiveness of the drivers. Some driving preferences of drivers can also be reflected in the figure. For example, compared with other drivers, driver Q01868D have high ranking of driving patterns “222” and “444.” The ranking of risk driving behavior patterns such as rapid acceleration and deceleration and the amplitude of acceleration and deceleration fluctuation can reflect the driver's driving behavior and potential danger, but some drivers with a more stable overall style also have risk driving behavior patterns. That is, drivers in the relative safety group had more risk driving behavior patterns (e.g., “000”) than those in the relative safety group. In addition, the low proportion of rapid acceleration and deceleration in the overall driving behavior does not mean that the driver's driving style is stable. It is necessary to judge the driver's driving style by combining the type and distribution of specific driving behavior patterns. It also illustrates the importance of judging individual drivers' driving styles.

### 4.4. Accelerated Driving Behavior

As can be seen from Figures 5 and 6, each chart represents the ranking from high to low of the occurrence frequency of the corresponding driver's accelerated driving pattern. The acceleration pattern diagram represents the similarities and differences and preferences of each driver in the acceleration pattern he or she chooses when taking the accelerated driving behavior. As can be seen from the figures, the occurrence frequency and ranking of the fast accelerating driving patterns defined as dangerous drivers, such as “555,” “666,” are generally higher than those of safe drivers. However, some safe drivers ranked higher than dangerous drivers in the accelerated driving pattern (e.g., mode “666”). For another example, for driver F63030, his rapid acceleration and deceleration frequency is not high in the proportion of the overall driving behavior, but the driver's preference in acceleration is relatively aggressive. This shows that the overall proportion of risk driving behavior can only reflect the driver's driving risk on one hand. The reason is that the increase of the frequency of safe driving mode will reduce the overall frequency proportion of some risk driving modes, leading to the concealment of some risk driving behaviors. Some drivers generally have a smooth driving style but are prone to violent driving behavior at certain moments. Although the frequency of these risk driving behaviors is not high, the problem of increasing accident probability caused by these behaviors cannot be ignored, which reflects the tendency of risk driving behaviors of drivers. Rankings and frequencies can complement each other to accurately differentiate the driving styles of different drivers.

It can be seen from the acceleration patterns of several drivers who are defined as safe drivers that with the increase of safety degree (the decrease of the overall proportion of drivers' acceleration and deceleration behaviors), such as “555,” “666,” the occurrence frequency and ranking of this dangerous pattern significantly decreased, and the acceleration behavior became more and more stable. In fact, in addition to the actual driving pattern occurrence frequency, the interaction between the “555” and “666” patterns and other patterns may also affect the driver's driving safety level. In addition, the degree of driving safety is determined by acceleration and deceleration behavior, not just acceleration.

### 4.5. Decelerated Driving Behavior

As can be seen from Figures 7 and 8 for the occurrence frequency of the driver's deceleration driving behavior pattern, the deceleration driving behavior pattern diagram represents the similarities and differences and preferences of each driver in the deceleration driving behavior. The pattern “000” and deceleration patterns with large acceleration variations are good indicators of the driver's style in deceleration driving behavior. The presumed danger group ranked higher in the “000” patterns, and some of their driving patterns reflected how hard they drove when slowing down. Drivers assumed to be in the safety group also experienced sharp deceleration patterns, such as mode “000,” but were generally more stable. It should be noted that the deceleration driving behavior pattern of B67845 and F63030 in the safety group indicates that their deceleration driving behavior is risky. The reason is that the driving pattern “000” ranks high, and there is a more aggressive driving pattern with large acceleration fluctuation. The F63030, in particular, was even more aggressive than some dangerous drivers in slowing down. In the previous two parts, it is also mentioned that the driver's integrated acceleration and deceleration behavior is not much, but in the face of acceleration and deceleration driving behavior, the driver's aggressive style, there is a potential accident risk. According to the deceleration pattern of different drivers, the driving preference and possible risk of each driver can be judged better.

### 4.6. Driver Acceleration Level Distribution

In order to further explore the acceleration preference adopted by drivers in acceleration and deceleration behavior, this section excludes drivers' uniform driving behavior (acceleration level 3) and calculates the proportion of acceleration and deceleration behavior of each level in the integrated acceleration and deceleration behavior. Based on the radar chart, the behavior data of different drivers are visually evaluated, and the results are shown in Figures 9 and 10.

The hexagons of the radar map represent different levels of acceleration. Level 3 is removed here to exclude the influence of a large number of uniform driving behaviors on the acceleration and deceleration behavior proportion. The percentages of each driver's different levels of acceleration are shown on the radar chart. The radar map clearly shows drivers' preferences at various levels of acceleration. It can be found from the radar maps of the two groups that the occurrence ratio of dangerous group drivers is generally higher than that of safety group drivers for the more severe acceleration behavior (acceleration level 6) and the more severe deceleration behavior (acceleration level 0). For acceleration level 5 and acceleration level 1, the average proportion of drivers in the danger group was higher than 10% and close to 15%. The safety group averaged closer to 10 percent. The distribution in the figure shows that the acceleration and deceleration behaviors of drivers in the safety group are generally more gradual than those in the dangerous group. However, there are certain exceptions in each group. The acceleration and deceleration behaviors of drivers F63030 in the safety group were extreme, with more slight acceleration and deceleration behaviors (grade 4 and grade 2) and severe acceleration and deceleration behaviors (grade 6 and grade 0), which were reflected in the figure as hourglass. The acceleration and deceleration behaviors of drivers in the dangerous group Q01868D also tended to moderate, especially the slight deceleration.

### 4.7. The Influence of Road Administrative Grade on Driving Behavior Pattern

Road administrative grade has a certain influence on the driving speed and acceleration and deceleration behavior of drivers. In order to further explore the influence of road administrative grade on drivers' driving behavior, this study selected a driver who had roughly the same driving time in the three road grades of national highway and above, provincial highway, prefectural highway, and below as a case to analyze. The driving behavior patterns of the driver under three different road administrative levels were compared, as shown Figure 11.

With the improvement of road administrative grade, the driver's driving behavior becomes more stable; that is, the relatively safe driving mode ranks higher and occurs more frequently. The driving behavior pattern with higher potential risk occurred more frequently and ranked lower. For example, in driving mode “000,” it can be clearly seen that as the administrative level of the road is lowered, the driving mode's ranking keeps rising. Driving pattern “000” is a typical driving behavior pattern with certain characteristics, which reflects the driver's driving preferences and habits. Under the conditions of three different administrative levels of roads, the driving patterns (e.g., driving pattern “000”) with individual characteristics of drivers all appear, but the ranking of the modes in their respective road conditions is different. This also reflects that the driver's driving style is relatively fixed and he can maintain his own driving style in different road conditions. The driving behavior pattern diagram can not only show the distribution of driving behavior, but also clearly present the driving styles and driving risks of drivers under different road grades. Compared with the traditional method of fixed threshold, the driving behavior pattern diagram can avoid the problem that the fixed threshold is not suitable for drivers in different situations and can show the driver's unique driving habits without being influenced by the environment.

### 4.8. Quantitative Assessment of Driving Risk

The driving behavior of drivers was comprehensively evaluated by the comparative evaluation model of driving risk. This section divides the driver's driving behavior into three parts: overall driving behavior score, accelerated driving behavior score, and decelerated driving behavior score.

As can be seen from Figure 12, the scores of different behaviors of different drivers reflect the level of drivers. The higher the score, the higher the risk of driving behavior, and the lower the comfort and economy of driving. In general, the scoring trend of different drivers is roughly the same as the ranking trend of drivers' behavior scale graph based on fixed threshold. Drivers with a high proportion of risk driving behavior scored higher on acceleration, deceleration, and overall driving behavior. Those who drove more consistently, with less risky driving, tended to have lower scores. But there are some exceptions. The two drivers, B32781 and B32791, had a high proportion of overall risk driving behaviors, but their overall evaluation score was low. According to the data, this is because the driving behavior patterns of these two drivers are scattered, and the proportion of the first 30 typical driving patterns in the overall driving pattern is lower than that of other drivers, resulting in a lower score. The reason why the driving behavior evaluation score chart and the driving behavior ratio chart based on the threshold are not completely consistent is that there is still a lack of a clear definition of potential risks in the safety analysis of driving behavior. This method can describe the driver's personalized driving behavior characteristics, comprehensively consider three factors of vehicle safety, driving comfort, and fuel economy, and quantitatively evaluate and compare the driver's driving risk.

In addition, the overall driving behavior score was different from that of only acceleration or deceleration. This is due to the difference in the pattern structure and frequency, and some drivers have more acceleration behavior or deceleration behavior. This phenomenon is acceptable. As can be seen from the figure, there are similar trends in the scores of these three behaviors among different drivers.

## 5. Discussion and Conclusion

According to the positioning data in the Internet of HDVs platform environment, this paper proposes an approach to evaluate the driver's driving risk and driving style with undefined threshold. Based on the vehicle driving data and the time series change of driver's driving behavior, the driving behavior pattern diagram was established. Through the driving behavior pattern diagram and driving risk modeling evaluation, the personalized driving behavior risk of different drivers was quantitatively evaluated, and the driving styles of different drivers were qualitatively and quantitatively compared. The main work and conclusions of this paper are as follows:

1. A graphic qualitative and quantitative analysis of individual driving behavior is carried out based on the change of driving behavior time series. Based on the positioning data of the actual HDVs, the driving behavior pattern was established to evaluate the driving behavior style and safety degree. The method is to evaluate the undefined threshold of the driver's driving style. Based on the vehicle driving data, a driving behavior pattern was established by using the driver's driving behavior changing with time.
2. Based on the driving behavior pattern diagram, the driving style of drivers is analyzed and evaluated qualitatively and quantitatively. The evaluation results show that the driving behavior pattern can reflect the driver's driving habits and potential risks. The ranking of risk driving behavior patterns such as rapid acceleration and deceleration and the amplitude of acceleration and deceleration fluctuation can reflect drivers' driving habits and risks. Drivers with a more stable overall style also have some risk driving patterns. It is necessary to judge the driver's driving style by combining the type and distribution of specific driving modes. Even less risk driving behaviors may lead to the occurrence of driving accidents, and these risk driving behaviors are easy to be hidden by the overall driving data. Drivers will have different preferences in the degree of acceleration and deceleration of their driving behavior when faced with acceleration or deceleration. The driver's acceleration grade distribution also further reflects the driver's driving habit and style. In general, drivers with a low proportion of rapid acceleration and deceleration will adopt more moderate driving behavior and lower acceleration level in the face of acceleration and deceleration. The driving behavior pattern diagram can reflect the distribution of driving behavior and clearly present the driving style, habits, and driving risks of drivers.
3. According to the frequency and ranking of typical driving modes of drivers, a risk assessment modeling method for driving behavior was proposed from three aspects of vehicle safety, driving comfort, and fuel economy, and the similarities and differences of driving behaviors of different drivers were quantitatively analyzed. The evaluation results show that drivers with a high proportion of risk driving behavior scored higher on acceleration, deceleration, and overall driving behavior. Those who drove more consistently, with less risky driving, tended to have lower scores. But there are some exceptions.

## Figures and Tables

**Figure 1:** Driving behavior pattern diagram.

**Figure 2:** Overall proportion of drivers' risk driving behavior.

**Figure 3:** Dangerous group driving behavior pattern diagram.

**Figure 4:** Safety group driving behavior pattern diagram.

**Figure 5:** Dangerous group driving behavior pattern diagram.

**Figure 6:** Safety group driving behavior pattern diagram.

**Figure 7:** Dangerous group driving behavior pattern diagram.

**Figure 8:** Safety group driving behavior pattern diagram.

**Figure 9:** Acceleration rating of dangerous group drivers.

**Figure 10:** Acceleration rating of safe group drivers.

**Figure 11:** Patterns of driving behavior under three administrative levels of roads.

**Figure 12:** Driving behavior evaluation score.

## Data Availability

The data used in this paper were collected by the information acquisition equipment installed on the HDVs. The collection device includes a GPS module for collecting location data, an OBU module for collecting vehicle movement data, and a cellular network.
